The article "URB597 and Andrographolide Improve Brain Microvascular Endothelial Cell Permeability and Apoptosis by Reducing Oxidative Stress and Inflammation Associated with Activation of Nrf2 Signaling in Oxygen-Glucose Deprivation" was published in 2022. Journal: Oxid Med Cell Longev.

# URB597 and Andrographolide Improve Brain Microvascular Endothelial Cell Permeability and Apoptosis by Reducing Oxidative Stress and Inflammation Associated with Activation of Nrf2 Signaling in Oxygen-Glucose Deprivation

**DOI:** 10.1155/2022/4139330

**Published:** 2022-05-12

**Authors:** Da-Peng Wang, Kai Kang, Jun Sun, Qi Lin, Qiao-Li Lv, Jian Hai

**Affiliations:** ^1^Department of Neurosurgery, Tong Ji Hospital, School of Medicine, Tong Ji University, Shanghai 200065, China; ^2^Department of Research and Surveillance Evaluation, Shanghai Center for Health Promotion, Shanghai 200040, China; ^3^Department of Pharmacy, Institutes of Medical Sciences, Shanghai Jiao Tong University School of Medicine, Shanghai 200025, China; ^4^Department of Head and Neck Surgery, Jiangxi Key Laboratory of Translational Cancer Research, Jiangxi Cancer Hospital, Nanchang University, Jiangxi 330029, China

## Abstract

Ischemic stroke, a cerebrovascular disease worldwide, triggers a cascade of pathophysiological events, including blood-brain barrier (BBB) breakdown. Brain microvascular endothelial cells (BMECs) play a vital role in maintaining BBB function. The injury of BMECs may worsen neurovascular dysfunction and patients' prognosis. Therefore, uncover the principal molecular mechanisms involved in BBB disruption in stroke becomes pressing. The endocannabinoid system (ECS) has been implicated in increasingly physiological functions, both in neurometabolism and cerebrovascular regulation. Modulating its activities by the fatty acid amide hydrolase (FAAH) shows anti-inflammatory characteristics. Andrographolide (AG), one Chinese herbal ingredient, has also attracted attention for its role in immunomodulatory and as a therapeutic target in BBB disorders. Recently, the FAAH inhibitor URB597 and AG have important regulatory effects on neuronal and vascular cells in ischemia. However, the effects of URB597 and AG on BMEC permeability and apoptosis in oxygen-glucose deprivation (OGD) and the underlying mechanisms remain unclear. To address these issues, cultured BMECs (bEnd.3 cells) were exposed to OGD. The cell viability, permeability, tube formation, and apoptosis were assessed following treatment with URB597, AG, and cotreatment. Mitochondrial membrane potential (MMP), reactive oxygen species (ROS), superoxide dismutase (SOD), catalase (CAT), malondialdehyde (MDA), proinflammatory factors, tight junction (TJ) proteins, and oxidative stress-mediated Nrf2 signaling were also investigated. Results revealed that OGD broke the endothelial barrier, cell viability, MMP, and tube formation, which was reversed by URB597 and AG. OGD-induced enhancement of ROS, MDA, and apoptosis was reduced after drug interventions. URB597 and AG exhibited antioxidant/anti-inflammatory and mitochondrial protective effects by activating Nrf2 signaling. These findings indicated that URB597 and AG protect BMECs against OGD-induced endothelial permeability impairment and apoptosis by reducing mitochondrial oxidative stress and inflammation associated with activation of Nrf2 signaling. URB597 and AG showing the vascular protection may have therapeutic potential for the BBB damage in ischemic cerebrovascular diseases.

## 1. Introduction

Ischemic stroke with a high rate of morbidity and mortality is becoming the major cause of adult long-term disability worldwide [1]. In stroke, there is not enough blood supply to provide nutrients and oxygen to ischemic zones, triggering a series of pathophysiological changes, such as inflammatory response, ischemia and hypoxia, and blood-brain barrier (BBB) leakage. BBB dysfunction is a critical neurovascular damage process, which devotes to hemorrhagic transformation and poor prognosis in patients [2]. The BBB is composed of three cellular elements, namely, glial end-feet, pericytes, and brain microvascular endothelial cells (BMECs) [3]. BMECs play a vital part in maintaining the structural and functional integrity of BBB, whereas disruption of microvascular can be found in ischemic cerebrovascular diseases [4]. How do BMECs respond to ischemia and hypoxia in an in vitro model of stroke (oxygen-glucose deprivation, OGD), as well as the underlying mechanisms involved in BBB impairment, remains confusing.

The endocannabinoid system (ECS) comprises endogenous cannabinoid receptors 1 and 2 (CB1 and CB2), the two endocannabinoid ligands N-arachidonoylethanolamine (anandamide, AEA) and 2-arachidonoylglycerol (2AG), and endocannabinoid anabolic and catabolic enzymes, such as monoacylglycerol lipase and fatty acid amide hydrolase (FAAH) [5]. The ECS is involved in modulating neural development, synaptic plasticity, endothelium-dependent vasorelaxation, cerebrovascular regulation, microvascular endothelial barrier, and BBB function [6]. The effects of the ECS on cardiovascular and cerebrovascular cells and circulatory system are not only by CBs but also other atypical cannabinoid receptor-manners. Mestre et al. have found that endocannabinoid (AEA) reduces leukocyte transmigration in a model of BBB by inhibiting vascular cell adhesion molecule-1 in brain endothelial cells associated with CB1 activation [7]. In ischemia-reperfusion injury, pharmacological CB2 offers a new strategy for the protection of blood-spinal cord barrier permeability [8]. The ECS may importantly modulate BBB function under physiological and pathophysiological conditions in a very complex manner. Nevertheless, the underlying pathophysiological characteristics are poorly understood. FAAH inhibitors can also upregulate the level of ECS, which improves ischemic neuronal and vascular injury. FAAH inactivation is emerging as a potential strategy to treat stroke [9]. However, the possible effects of FAAH inhibitors on BMECs as well as BBB permeability during OGD have not yet been systematically investigated.

Andrographolide (AG) is a major active compound of the Asian herb plant *Andrographis paniculate* (green chiretta), which possesses diverse biomedical effects including antineoplastic, antibacterial, anti-inflammatory, and antioxidant properties [10]. Growing evidence indicates that AG with the beneficial neurofunctional regulation exhibits therapeutic effects in Alzheimer's disease (AD) and ischemic brain damage [11]. AG can reduce the total A*β* burden in aged Octodon degus [12]. And we previously reported that AG could suppress cerebral ischemia-induced hippocampal neuronal apoptosis and astroglial activation [13, 14]. Recently, the effects of AG on BBB permeability in ischemic stroke gained attention. Pharmacodynamic studies have revealed that AG can cross the BBB and protect against the MCAO-induced primary cerebral endothelial cells injury [15], but the underlying mechanisms remain unclear.

To clarify these issues, in this study, we explored the potential effects of FAAH inhibitor URB597 and AG on mice BMECs (bEnd.3 cells), as well as the underlying mechanisms associated with its therapeutic potential in modulating BBB permeability in OGD.

## 2. Materials and Methods

### 2.1. OGD Treatment

To mimic cerebral ischemia in vitro, bEnd.3 cells (No. CL-0598, Procell Life Science & Technology Co., Ltd, Wuhan, China) were exposed to OGD as reported previously [16]. Briefly, cells were cultured in RPMI 1640 medium (Gibco, Herndon, USA) containing 10% fetal bovine serum (Gibco, Herndon, USA), 100 U/mL penicillin, and 100 U/mL streptomycin (Hyclone Laboratories, Logan, USA) in a humidified incubator at 37°C with 5% CO_2_ and 95% air. Then, cells were transferred from the RPMI 1640 medium to DMEM without glucose (Gibco, USA) in 6-well plates, then subsequently cultured in a humidified incubator at 37°C with 5% CO_2_ and 95% N_2_ for 24 hours.

### 2.2. Experimental Groups and Drug Treatment

To assess the effects of OGD on bEnd.3 cells and choose the optimum duration of OGD, the cell viability was measured after 4-24 h of OGD in bEnd.3cells. For drug concentration screening, URB597 and AG (No. HY-10864, No. HY-N0191, Med Chem Express Co., Ltd, Shanghai, China) were dissolved in dimethylsulfoxide (DMSO, Med Chem Express, Shanghai, China) and diluted with serum-free RPMI 1640 at different concentrations (0.5 *μ*M, 1 *μ*M, 2 *μ*M, 5 *μ*M, and 10 *μ*M), respectively. Then, cells were added with different concentrations of URB597 and AG before OGD treatment. After 6 h of OGD, cells were incubated in a maintenance medium for 12 h under normal conditions subsequent experiments. Experimental treatment groups were as follows: (1) the control group was cultured without OGD exposure (the Con group), (2) the OGD treatment (the OGD group), (3) the URB597 (2 *μ*M) treatment during OGD (the URB group), (4) the AG (10 *μ*M) treatment during OGD (the AG group), and (4) the URB597 and AG cotreatment during OGD (the URB + AG group).

### 2.3. Cell Viability Assay

A 3-(4,5-dimethyl-2-thiazolyl)-2,5-diphenyl-2-H-tetrazolium bromide (MTT) method was used to assay cell viability. In brief, the cells in different groups were incubated for another 4 h at 37°C and 5% CO_2_ in a sterile incubator, following added 20 *μ*l of MTT. The supernatant was removed, and the cells were lysed in 150 *μ*l of DMSO. A microplate reader (Epoch, BioTek, USA) was used to measure the absorbance (OD) at 490 nm. Cell viability was expressed as a percentage of the control [17].

### 2.4. LDH Leakage Assay

LDH release was detected using the LDH activity kit (Beyotime, Shanghai, China) as previously described [18]. Briefly, 50 *μ*l supernatant from each sample was transferred into a new plate, mixed with 50 *μ*l kit's reaction mixture, and incubated for 10 min at room temperature. Stop solution was then added. The OD values at 490 nm and 630 nm were measured using a microplate reader (Epoch, BioTek, USA).

### 2.5. The Tube Formation Assay

For tube formation analysis, Matrigel basement membrane matrix with growth factor-reduced (BD Biosciences, San Jose, CA, USA) was used as previously described [19]. First, the matrix was thawed at 4°C overnight and incubated at 37°C for 30 mins [20]. After Matrigel polymerization, the pretreated bEnd.3 cells were resuspended and seeded onto the primary Matrigel (60 *μ*l). The plate was transferred to a humidified incubator for 12 h incubation. Images were taken using a microscope (Olympus, Tokyo, Japan) with magnification at ×40 from 3 randomly selected optical fields. The tube formation assay was analyzed and interpreted by an experimenter blinded to the details of the study using the Wim Tube software (Wimasis, Munich, Germany). The number and length of the capillary-like tube were quantified.

### 2.6. Brain Microvascular Endothelial Barrier Permeability Assay

To estimate the integrity of the cell monolayer, transendothelial electrical resistance (TEER) was first measured using a Millicell-Electrical Resistance System (Millipore, Bedford, MA) with an electrode as described previously [17]. One electrode was put into the upper Transwell insert compartment, and the other electrode was inserted into the lower compartment inside a cell culture hood at room temperature [21]. The resistance was measured daily at regular intervals until cells reached a consistent resistance. Triplicate measurements were recorded for each monolayer with values expressed as *Ω* cm^2^.

Brain microvascular endothelial barrier permeability was also tested using the flux of Evans blue (EB) dye-labeled albumin (Sigma, MU, USA) across the cell monolayer. EB-albumin (50 *μ*l of 2% concentration) was added to the apical surface of bEnd.3 cell monolayers in the culture insert for 1 h before the end of the OGD, whereas bovine serum albumin (150 *μ*l of 4% concentration) was added to the lower chamber. The media in the lower chamber was collected to detect the absorbance of EB at the wavelength of 630 nm using a microplate reader (Epoch, BioTek, USA), after incubation at 37°C for 1 h.

### 2.7. Oxidative Stress Assay

Intracellular oxidative stress was evaluated by using the determination of superoxide dismutase (SOD), catalase (CAT), malondialdehyde (MDA), and the 2,7-dichlorofluorescein diacetate (DCF-DA) with commercial kits (Beyotime, Shanghai, China) [16]. Experiments were performed in 96-well plates for each condition at least in triplicate. For the ROS assay, cells were incubated with 5 *μ*M DCF-DA solution at 37°C and 5% CO_2_ for 30 mins, after being centrifuged at 1000 rpm for 5 min and washed twice with PBS. Then, the mean fluorescence intensity (MFI) was evaluated using a fluorometric microplate reader (FilterMax F5, Molecular Devices, Sunnyvale, USA). The excitation and emission wavelengths were set at 485 and 535 nm, respectively.

### 2.8. Mitochondrial Membrane Potential (MMP, *Δψ*m) Measurement

According to the instruction of the JC-1 kit (Beyotime, Shanghai, China), cells were plated in 96-well plates at a density of 1 × 10^4^/well after 24 h treatment for measuring *Δψ*m. In brief, the cells were washed twice with PBS and incubated with JC-1 staining medium (2 *μ*M) at 37°C for 20 mins. The cells were observed under a fluorescence microscope (Zeiss, Jena, Thuringia, Germany) after washing with PBS. The level of cellular red and green fluorescence was analyzed by Image J (NIH, Bethesda, MD). Values are expressed as the rate of the red/green fluorescence intensity by an investigator blinded to the grouping information.

### 2.9. q-Reverse Transcription-Polymerase Chain Reaction (qRT-PCR)

The total RNA of BMECs was obtained by using the TRIzol reagent. The RNA concentration and purity were detected by using a Nanodrop Spectrophotometer (ND-100, Thermo, Waltham, MA) at the 260/280 nm ratio. The total RNA was dissolved in 10 *μ*l DEPC-treated water. The reverse transcription and cDNA production were performed by using a PrimeScript RT reagent kit (RR047A, Takara Holdings Inc., Tokyo, Japan) according to the manufacturer's protocol. The cDNA fragment was amplified by PCR using the following specific primers: TNF-*α* forward: 5′-CAT CTT CTC AAA ATT CGA GTG ACA A-3′, reverse: 5′-TGG GAG TAG ACA AGG TAC AAC CC-3′; IL-1*β* forward: 5′-TCA TTG TGG CTG TGG AGA AG-3′, reverse: 5′-AGG CCA CAG GTA TTT TGT CG-3′; iNOS forward: 5′-GAC GAG ACG GAT AGG CAG AG-3′, reverse: 5′-CAC ATG CAA GGA AGG GAA CT-3′; *β*-actin forward: 5′-TGT GAT GGT GGG AAT GGG TCA G-3′, reverse: 5′-TTT GAT GTC ACG CAC GAT TTC C-3′. The expression of specific mRNAs was validated by performing quantitative real-time PCR with One-Step SYBR PrimeScript RT-PCR Kit (Perfect Real Time, RR066A, Takara Bio Inc., Japan). The relative gene expression level was evaluated by using the 2-*ΔΔ*Ct method, which was normalized to endogenous GAPDH expressions.

### 2.10. Western Blot Analysis

The total protein of BMECs was extracted by using RIPA buffer (Beyotime, Shanghai, China). The protein samples were quantified via a BCA assay kit (Beyotime, Shanghai, China). Subsequently, 30 *μ*g protein in each group was separated by using SDS-PAGE and transferred onto 0.45 *μ*m polyvinylidene fluoride (PVDF) membranes (Millipore, MA, USA). The membranes were blocked in 5% skim milk. Next, the membranes were incubated overnight with primary antibody against ZO-1 (1 : 1000, ab221547, Abcam, Cambridge, MA, USA), Occludin (1 : 1000, ab216327, Abcam), Claudin 5 (1 : 1000, ab131259, Abcam), Nrf2 (1 : 1000, bs-1074R, Bioss, Beijing, China), and HO-1 (1 : 1000, ab52947, Abcam) at 4°C and then interacted with secondary antibody for 2 hours. Protein bands were revealed by the enhanced chemiluminescence (ECL) method. *β*-Actin (1 : 5000, Abcam, ab227387) was used as a loading reference.

### 2.11. Flow Cytometry Analysis

To estimate the proportions of apoptosis cells, cellular sedimentation was measured by using flow cytometry. After treatment, the BMECs were detached with 0.25% trypsin containing no EDTA (Thermo Fisher) and then centrifuged at 3000 rpm, after which the supernatant was discarded. The cells were resuspended in PBS, centrifuged, and with the supernatant removed again. The cell apoptosis was quantified by using the Annexin V Apoptosis Detection kit (K201-100; BioVision, Milpitas, CA, USA). The Annexin-V-FITC/PI staining solution was compounded by HEPES buffer (Thermo Fisher), Annexin-VFITC/PI (50 : 1 : 2). The cells were resuspended with the prepared dye at 100 *μ*l per tube. And the tube was protected from light. After incubating for 15 min at ambient temperature, the cells were lysed with 1 mL HEPES buffer. Finally, the cells were collected into flow tubes, and the cell apoptosis was measured on the flow cytometer at 488 nm (Epoch, BioTek, USA).

### 2.12. Immunofluorescence Staining

Immunofluorescence staining was used to detect the expression of vWF (No. sc-365712, Santa Cruz Biotechnology, Dallas, Texas, USA), ZO-1, Occludin, and Nrf2. First, using 4% paraformaldehyde, fix the cells at room temperature for 10 minutes then washing twice in PBS. Next, the cells were permeabilized in Triton X-100 solution (0.5% TritonX-100 dissolved in PBS) for 30 minutes and treated with 5% bovine serum albumin (BSA) in PBS for 30 minutes. After removal of the blocking solution, cells were incubated with rabbit anti-ZO-1, Occludin, and Nrf2 monoclonal antibody at 1 : 200 dilution in 5% BSA overnight at 4°C. Subsequently, fluorescent dye-conjugated secondary antibody was added and incubated with the cells for 2 hours away from light. Finally, the immunofluorescence images were examined using a fluorescent microscope. The mean fluorescence intensity was estimated from 4 fields of view in each sample by an investigator without knowing the treatment.

### 2.13. Terminal Deoxynucleotidyl Transferase dUTP Nick End Labeling (TUNEL) Assay

Cells were plated in 24-well flat-bottomed plates at a density of 1 × 105 cells per well, fixed with 4% paraformaldehyde for 30 minutes, and then permeabilized by 0.2% TritonX-100 for 5 minutes. The apoptosis levels were detected by using Apoptosis Detection Kit (RiboBio, China). Adding 50 *μ*L of TUNEL detection solution to each well and incubating for one hour at room temperature in the dark. The numbers of TUNEL-positive cells were observed under a fluorescence microscope (Olympus).

### 2.14. Small Interfering RNA (siRNA) Transfection

Nrf2 siRNA was purchased from RiboBio Co., Ltd. (siG2006160258184354, RiboBio, Guangzhou, China). Transfection of negative control (NC) siRNA and Nrf2 into BMECs with Lipofectamine 3000 (Thermo Fisher, UT, USA) is according to the manufacturer's instructions. Cells were then harvested 72 hours later for Western blotting to assess the expression of Nrf2 and HO-1.

### 2.15. Statistical Analysis

All data, presented as the mean ± standard error of the mean (SEM), were analyzed by two technicians blinded to the details of the group using SPSS 22.0 software (IBM, USA) and GraphPad Prism 6.0 software (San Diego, CA). The student's *t*-test was used for comparison between two groups. One-way analysis of variance (ANOVA) followed by a Bonferroni post hoc test was used for comparison among multiple groups. A *p* value less than 0.05 was considered statistically significant for all tests.

## 3. Results

### 3.1. The Effects of Different Concentrations of URB597 and AG on the Viability of bEnd.3 Cells in OGD

As shown in Figure 1(a), cells were examined for morphology and growth status and identified by immunofluorescence stain of vWF. Then, we investigated the deleterious effects of different durations of OGD on the viability of bEnd.3 cells using MTT assay. As time went on, the viability of cells deteriorated (Figure 1(b)). The viability of cells significantly decreased in the OGD 6 h compared with the control, which is approximately 60.2% of the control. The viability of the cell was reduced more than 50% after 12 h and 24 h of OGD. Then, the bEnd.3 cells were treated with URB597 (C_20_H_22_N_2_O_3_) and AG (C_20_H_30_O_5_) at different concentrations (0.5 *μ*M, 1 *μ* M, 2 *μ*M, 5 *μ*M, and 10 *μ*M) subjected subsequently to 6 h of OGD (Figures 1(c) and 1(d)). As shown in Figure 1(c), URB597 (2 *μ*M and 5 *μ*M) treatment increased the viability of cells compared with the OGD. On the contrary, the URB597 treatment with higher concentration led to the viability of cells decreased. 5 *μ*M and 10 *μ*M of AG treatment protected 72.6% and 84.3% of the cells, respectively. The results indicate that URB597 with the concentration of 2 *μ*M and AG with the concentration of 10 *μ*M are propitious to bEnd.3 cells subjects to OGD.

### 3.2. URB597 and AG Increase the Viability of bEnd.3 Cells in OGD

To further determine whether URB597 treatment, AG treatment, as well as cotreatment promote cell growth and survival under conditions of OGD, we assessed the fluorescence staining of vWF (Figure 2(a)). After 6 h of OGD, vWF fluorescence intensity was significantly reduced (*p* < 0.05 vs. Con). However, URB597 treatment and AG treatment significantly increased the expression of vWF (all *p* < 0.05, vs. OGD group). Compared with the fluorescence intensity of vWF in the URB group and the AG group, vWF expression is higher in the URB + AG group (all *p* < 0.05) (Figure 2(b)). In the MTT assay, OGD caused a decline in cell survival and growth with OD values decreasing during culture, which was reversed in the drug intervention groups (Figure 2(c)). In addition, LDH leakage as a marker for cell degradation was also monitored. As shown in Figure 2(d), LDH leakage increased in the OGD group compared with the control group (*p* < 0.05). URB597 (2 *μ*M) and AG (10 *μ*M) treatment significantly reduced it (all *p* < 0.05, vs. OGD group). Meanwhile, the inhibition is more obvious in cotreatment group (*p* < 0.05, vs. URB group; *p* < 0.05, vs. AG group). Taken together, these results suggested that UBR597 and AG increased the survival and growth of endothelial cells during OGD in vitro.

### 3.3. URB597 and AG Promote the Tube Formation in bEnd.3 Cells Subjected to OGD

Previous studies suggested that ECS and AG were involved in endothelial cell angiogenesis [22]. To further investigate the effects of URB597 and AG on the tube formation of BMECs, the total pipe length of the tube-like structure in bEnd.3cells that had been treated with URB597, AG, and both, was measured after 12 h of culture under OGD. At the beginning of the OGD (0 h), there are no differences were found among groups; however, the tube-like structure was different after 12 h of OGD (Figure 3(a)). Statistical results show that the total pipe length of the tube-like structure in the OGD group was significantly decreased compared to the cells in the Con group (*p* < 0.05). This reduction was reversed by pretreatment with URB597, AG, and combination (all *p* < 0.05, vs. OGD group) (Figure 3(b)). Thus, this result indicated that URB597 and AG treatments promote the tube formation of BMECs in OGD.

### 3.4. URB597 and AG Revert OGD-Induced Endothelial Barrier Leakage

The microvascular endothelial barrier is one important basis of the BBB, and its leakage was measured using TEER and EB-albumin assay. TEER, a measure of ion flux, was destroyed by OGD leading to declining over time [17]. The cell permeability was measured at 4 h of OGD, as the cell viability was not affected by OGD at that point (supplementary figure). As shown in Figure 3(c), the reduction of TEER induced by OGD was significantly improved by URB treatment (*p* < 0.05, vs. OGD group). A similar increment was found after treating with AG (*p* < 0.05, vs. OGD group). In the cotreatment group, the TEER was also raised.

Instead, with the opening of ion channels, the EB-albumin permeability significantly raised in OGD (*p* < 0.05, vs. Con group) (Figure 3(d)). URB treatment and AG treatment reduced the EB-albumin leakage. In addition, the EB-albumin level in the combination therapy group was lower levels than those in the URB group and the AG group (*p* < 0.05, respectively) and had the optimal effectiveness in suppressing endothelial barrier leakage (Figure 3(d)). These results above demonstrated that treatment with URB and AG reverted microvascular endothelial barrier leakage induced by OGD, showing the protective effect on endothelial cell permeability.

### 3.5. URB597 and AG Inhibit OGD-Induced Mitochondrial Oxidative Stress Inflammatory Response

Oxidative stress and inflammatory response are critical pathological processes in cerebral ischemia injury, and their intimate interactions mediate neuronal damage, endothelial cell permeability dysfunction, causing the accumulation of mitochondrial ROS [23]. We found that the level of ROS was upregulated in OGD cells (*p* < 0.05, vs. Con group) (Figures 4(a) and 4(b)). Compared with the control cells, proinflammatory factors' mRNAs, TNF-*α*, IL-1*β*, and iNOS, were upregulated in the OGD group (all *p* < 0.05) (Figures 4(c)–4(e)). In addition, cells in the OGD group presented decreased levels of SOD and CAT (*p* < 0.05, respectively, vs. Con group) and increased MDA (*p* < 0.05, vs. Con group) (Figures 4(f)–4(i)). Those elevated ROS, MDA, and inflammatory factors were inhibited by URB597 treatment, AG treatment, and cotreatment (all *p* < 0.05, vs. OGD group). Moreover, the cotreatment had the optimal effectiveness in antioxidation and anti-inflammation (all *p* < 0.05, vs. URB + AG group) (Figures 4(a)–4(i)). Therefore, these data showed that URB597 and GA inhibited OGD-induced mitochondrial oxidative stress and the resultant inflammatory response.

### 3.6. URB597 and AG Attenuate OGD-Induced MMP Injury

To determine whether ROS permeabilizes the mitochondrial membrane, MMP was measured using the cyanine dye JC-1. The accumulation of JC-1 in these organelles results in the formation of J-aggregates (high MMP, red fluorescence), which is in addition to the typical green fluorescence of J-monomers (low MMP) [24]. The decrease in the ratio between the red and green fluorescence intensity is a marker of mitochondrial damage. As shown in Figure 5, OGD led to a significant decrease in the MMP of BMECs (*p* < 0.05, vs. Con group). However, the decrease in OGD-induced MMP was notably alleviated in the URB group, the AG group, and the URB + AG group (all *p* < 0.05, vs. OGD group) (Figure 5(a)). In addition, URB597 combined with AG treatment was more effective than single treatment (*p* < 0.05, vs. URB + AG group) (Figure 5(b)). These findings confirmed that the URB597 and AG treatments attenuated OGD-induced mitochondrial depolarization, as they have synergistic protective effects on MMP in OGD.

### 3.7. URB597 and AG Upregulate the Expression of the Tight Junction (TJ) Proteins and Activate Nrf2 Signaling in OGD

The BBB is one of the most robust physical barriers, comprised of TJ proteins in BMECs [25]. We further investigated the effects of URB and AG on TJ membrane proteins, including ZO-1, Occludin, and Claudin 5, against OGD-induced injury. As shown in Figures 6 and 7, OGD led to decreasing expression of ZO-1, Occludin, and Claudin 5. After URB and AG treatment, the relative fluorescence intensity of ZO-1 and Occludin was elevated (all *p* < 0.05, vs. OGD group) (Figures 6(a)–6(c)). Western blot analysis revealed that ZO-1, Occludin, and Claudin 5 expressions were markedly reduced in the OGD group as compared to the Con group (all *p* < 0.05, vs. Con group) (Figures 7(c) and 7(e)–7(g)). These reductions were reversed by URB treatment, AG treatment, and cotreatment. Compared with the URB group or AG group, the upregulation effect of TJ proteins was the most significant in the URB + AG group (all *p* < 0.05) (Figures 6(b) and 6(c), Figures 7(e)–7(g)). These findings suggested that URB and AG could promote the expressions of ZO-1, Occludin, and Claudin 5 of BMECs in the condition of OGD.

To clarify the mechanism underlying the effects of URB and AG, we investigated changes in Nrf2 signaling in each group. The Nrf2 protein with the red fluorescence was mainly expressed in cytoplasm and nucleus (Figure 7(a)). OGD decreased the relative fluorescence intensity of Nrf2 level, which was reversed by URB treatment and AG treatment (all *p* < 0.05, vs. OGD group) (Figure 7(b)). More significant increase was found in the URB + AG group (*p* < 0.05, vs. URB group) (Figure 7(b)). Western blot analysis revealed that Nrf2 expression was downregulated by OGD (Figures 7(c) and 7(d)). However, URB treatment, AG treatment, and cotreatment increased the level of Nrf2 protein. In addition, compared with the siNC group, the levels of Nrf2 and HO-1 were deceased following siRNA silencing. However, the expression of Nrf2 as well as its downstream HO-1 was increased after URB597 and AG treatment, respectively (Figures 7(h)–7(k)) (*p* < 0.05, vs. siNrf2 group). All of these results suggested that URB597 and AG could upregulate the expression of TJ proteins and activate Nrf2 signaling in OGD.

### 3.8. URB597 and AG Suppress OGD-Induced Apoptosis

MMP and endothelial barrier impairment are hallmark events in triggering the early stage of energy deterioration, pathological changes, and cell apoptosis [26]. First, the cell apoptotic ratio was determined by TUNEL fluorescence staining (Figure 8(a)). The number of TUNEL-positive apoptotic cells with green fluorescence was very obvious in the OGD group (*p* < 0.05, vs. Con group). However, the URB597 treatment and the AG treatment significantly reduced the number of green fluorescent cells (all *p* < 0.05, vs. OGD group). Furthermore, the TUNEL-positive apoptotic cells continued to decrease in the cotreatment group compared with the URB group and the AG group (all *p* < 0.05) (Figure 8(b)).

To further confirm the antiapoptotic effect of URB597 and AG, we detected cell apoptosis by Annexin V-FITC/PI flow cytometry analysis. As shown in Figure 8(c), the apoptotic rate was 34.3 ± 2.2% in the OGD group, which was greatly increased compared with the control group (*p* < 0.05) (Figure 8(d)). Cells pretreated with AG and URB597 had a reduced apoptotic rate with 26.2 ± 1.7% and 24.5 ± 1.5%, respectively. The antiapoptotic effect of combined treatment was more effective than single treatment (*p* < 0.05, vs. URB + AG group) (Figure 8(d)). These results were consistent with the staining of TUNEL fluorescence. All of these findings suggested that URB597 combined with AG could mitigate OGD-induced TUNEL-positive cellar apoptosis levels better.

## 4. Discussion

BMECs form a barrier that is highly restrictive to the passage of solutes between nervous tissue and circulating blood [27]. It is a vital structure for maintaining BBB function and brain homeostasis that is vulnerably disrupted in various neurological diseases. Traumatic brain injury can, directly and indirectly, cause BMECs barrier rupture [28]. In an experimental animal model of stroke, cerebral ischemia destroys the BBB permeability, leading to an increase of brain EB content and brain water content [29]. In the present study, microvascular endothelial barrier function is disrupted in OGD, showing the TEER decline. TEER, a strong indicator of the integrity of the cellular barriers, is inversely related to the fractional area of pathways open to water and small molecules across a cell monolayer [30]. One potential mechanism for this decline is that OGD can open multiple ion channels, such as calcium ion channels [31]. We also found that EB leakage was increased by OGD, which is in line with previous reports [32]. Furthermore, BBB microvascular network is developed via vasculogenesis [33]. In cell viability and tube formation assay, the cellular activity and the length of a tubular structure in the OGD group were significantly decreased. These data demonstrate that OGD destroys the endothelial growth and barrier function, causing increased permeability of BMECs.

Biochemical characteristics of BBB damage include decreased expression and altered organization of TJ constituent proteins [4]. To evaluate the changes of TJ structural and regulatory proteins, we performed the fluorescence staining and western blotting for ZO-1, occludin, and Claudin-5. As shown in Figure 6, the lower immunostaining of ZO-1 and occludin together with the shift of intracellular localization of ZO-1 and occludin from the membrane to the cytoplasm in BMECs in the OGD group is indicating the altered TJ structures induced by OGD. In western blotting, OGD led to a significant reduction in levels of ZO-1, occludin, and Claudin-5 proteins. Since the frayed TJ structure has been shown to result in disruption of BBB integrity compared to intact TJ [34], likely, increased frayed TJ formations, as well as the decreased expression of TJ proteins in BMECs was, at least in part, causally implicated in permeability damage in OGD. In addition, endothelial barrier dysfunction involved in ischemic cerebrovascular pathogenesis may be a trigger, or consequence, of oxidative stress and inflammatory responses [35]. Here, a robust inflammatory response is activated by OGD with proinflammatory cytokine mRNA (TNF-*α*, IL-1*β*, and iNOS) upregulation, which is one of the most important mechanisms for cellular metabolism and barrier function disorder. As inflammation after stroke not only lead to the remodeling of TJ but also promote cellular ROS accumulating [36]. ROS were considered as one of the key factors in cellular damage and tissue injury. Mitochondria are the main organelles of cellular ROS production, which are necessary for numerous fundamental functions, including respiration and oxidative energy production, regulation of the intracellular homeostasis [37]. During OGD events, BMEC cannot utilize mitochondrial mechanisms that allow it to maintain normal energy and metabolism, that producing ROS and inflammatory factors in excess and even worse MMP dysfunction. MMP impairment further triggers a series of cascades, including mitochondrial permeability damage and cell apoptosis [38]. In this study, accumulation of ROS levels combined with an imbalance of oxidant and antioxidant enzymes (descended SOD and CAT, elevated MDA) is demonstrated in OGD. When the greater imbalance occurs in favor of the ROS, mitochondrial oxidative stress and BMEC barrier damage ensue.

URB597, a relatively selective inhibitor of FAAH, promotes activities of ECS by enhancing its ligand and receptor levels. ECS is a physiological system with the capacity to mitigate cardiovascular and cerebrovascular disorders through neuronal and endothelial actions [39]. In our previous study, URB597 showed neuroprotective effects on primary cultured hippocampal neurons against OGD-induced neuronal apoptosis by activating CB1-brain-derived neurotrophic factor signaling [16]. Furthermore, we recently found that URB597 could improve neurovascular unit damage via suppressing neuroinflammation and ROS in rats with chronic cerebral ischemia [40]. In this study, we have demonstrated that the novel vascular protective effects of URB597 are involved with anti-inflammation and antioxidation. Levels of ROS and proinflammatory cytokines were significantly decreased in URB597 treatment. OGD-induced mitochondrial MMP disruption was also prevented by URB597. Meanwhile, URB597 improved the BMECs permeability damage compared with that in the OGD group. The clear mitochondrial protective action combined with anti-inflammation and antioxidation is probably the key underlying mechanism for keeping the BMECs barrier. Indeed, basic research results accumulated since the late 1990s indicate that the moderating effects of ECS on vascular endothelium actualize via attenuating vascular inflammation [41]. ECS can regulate redox function at multiple levels, with a range of downstream effects of cells and tissues. In cardiovascular aging and atherosclerosis, FAAH knockout can decrease age-related cardiac dysfunction, myocardial nitrative stress, and inflammatory gene expression [42]. Another reason for this endothelial protection is that reduction of TJ proteins, ZO-1, Occludin, and Claudin 5, induced by OGD was reserved by URB597 treatment. For morphological evidence, URB597 is proven to reduce ultrastructural deterioration of TJ and improve capillary endothelium breakage and vague basal lamina in cerebral ischemia [40].

AG's ability to prevent or mediate neurodegeneration and oxidative stress in cerebral ischemia in vivo was confirmed [11, 13, 15]. However, the study of modulated effects of AG on BBB function in stroke in vitro or in vivo models has been reported rarely. Yen et al. have reported that AG modulates the oxidative stress-related signaling pathways in primary cerebral endothelial cells to provide positive protection against OGD, maintaining the integrity of the endothelial barrier [43]. In hCMEC/D3, AG-loaded nanoparticles improve the permeation of AG without damaging BBB [44]. In this study, AG ameliorates the permeability of BMECs at various inflammation-mediated mechanisms, including antioxidative stress, inhibition of proinflammatory factors, and protecting mitochondria under the condition of OGD. Like URB597, AG upregulates the expression of ZO-1, Occludin, and Claudin 5 and keeps restoration of BBB integrity. Interestingly, in URB597 and AG cotreatment, we find a novel biological action is that the AG and URB597 display the positive synergistic protective effect on BMEC permeability and survival. However, AG (at 50 and 100 *μ*M concentrations) was reported to induce cerebral endothelial cell apoptosis via arresting cell cycle at the G_0_/G_1_ phase in cerebral ischemia/reperfusion model in vitro [45]. The discrepancy between this result and ours can be explained by differences in the duration of OGD and the dosage of AG that were used. Both AG and URB597 have a favorable safety profile in a time-dependent and dose-dependent manner [10, 11, 46].

Nrf2, a member of the cap-n-collar family of basic leucine zipper proteins, is basically bound in the cytoplasm to Kelch-like ECH-associated protein 1 (Keap1), directing it to ubiquitination and subsequent degradation by the proteasome [47]. Activating Nrf2 signaling shows neuroprotection against cerebral ischemia by antioxidative stress and antiapoptosis [48]. A deficiency of Nrf2 protein has been observed in neurodegenerative diseases, vascular inflammatory disorders, and stroke [49]. Nrf2 knock-out mice with more serious cerebral infarction, inflammatory damages, and neurological deficits were found compared with wild-type mice [50]. Physiological and pharmacological actions of URB597 and AG in treating many diseases are related to the regulation of the Nrf2. There is a simultaneous increase in Nrf2 expression in the brain of rats with hypertension caused by intraperitoneal injection with URB597 [51]. AG attenuates neurovascular injuries induced by cerebral ischemia via activating Nrf2 signaling, inhibiting inflammatory response [43, 52]. In this OGD model of BMECs, both URB597 and AG enhanced Nrf2 expression and may further cause Nrf2 to translocate into the nucleus. That results in subsequently suppressing the transcription of downstream targets (HO-1), proinflammatory genes, and oxidative metabolism. Excessive ROS is the primary stimulus of vascular dysfunction, which generates large numbers of potentially harmful intermediates that cause imbalances between prooxidants and antioxidants in vascular endothelial cells [53]. Furthermore, the decreasing Nrf-2 and HO-1 following siRNA silencing was reversed by URB treatment and AG treatment, respectively. These findings reveal that the protective effects of URB597 and AG on OGD-induced BMEC barrier damage and apoptosis are associated with activation of the Nrf2 signaling cascade. In addition, the role of URB597 and AG in modulating the Nrf2 pathway may be related to the fact that both can inhibit nuclear factor kappa light chain enhancer of activated B cells (NF-ĸB) signaling. There is a complex cross-talk between the Nrf2 and NF-*κ*B pathway, and NF-*κ*B can modulate Nrf2 transcription and activity, whereas Nrf2 counteracts NF-*κ*B-driven inflammatory response [54].

There are some limitations to this study. Under stress conditions (excessive accumulation of ROS and inflammatory stress), Nrf2-Keap1 interaction is disrupted, and Nrf2 translocates into the nucleus encoding proteins (i.e., HO-1) that counterbalance impairments in inflammatory and redox control [55]. Therefore, it would be more helpful to confirm Nrf2 is mediating these vascular protective effects if nuclear translocation of Nrf2 was also accessed. Second, mitochondrial oxidative stress is accessed by testing the levels of ROS, SOD, CAT, and MDA, but mitochondrial-specific probes such as MitoSOX are more suitable for measurement of mitochondrial ROS than DCF-DA. In addition, our demonstration of endothelial barrier preservation would benefit from additional experiments, such as check the levels of the inflammatory cytokines by ELISA, Evans blue staining for BBB permeability, and transmission electron microscope for BBB ultrastructure in vivo. The limitations should be further improved in animal experiments.

To our knowledge, the present study demonstrates for the first time that the FAAH inhibitor URB597 and AG protects BMECs against OGD-induced permeability impairment and apoptosis (proposed mechanism of URB and AG shown in Figure 9). This vascular protection is closely associated with activation of the Nrf2 signaling as well as anti-inflammatory and antioxidative effects, providing a new potential strategy for the treatment of endothelial barrier damage in ischemic cerebrovascular diseases.

## Figures and Tables

**Figure 1:** Effects of URB and AG on the cell viability of BMECs subjected to OGD. (a) Morphology and fluorescent staining of BMECs. (b) The cell viability was measured after 4–24 h of OGD by MTT. (c, d) The cell viability was measured after being treated with URB597 and AG (0.5 *μ*M, 1 *μ*M, 2 *μ*M, 5 *μ*M, and 10 *μ*M) subjected subsequently to 6 h of OGD by MTT. ^∗^*p* < 0.05, ^∗∗^*p* < 0.01*ν*s. Con, ^#^*p* < 0.05*ν*s. OGD, (*n* = 6).

**Figure 2:** Effects of URB and AG on the cell growth and LDH release of BMECs subjected to OGD. (a, b) Representative vWF (green) immunofluorescence for BMECs. (c, d) Statistical analysis of the cell viability (MTT method) and LDH release. ^∗^*p* < 0.05, *ν*s. Con, ^#^*p* < 0.05*ν*s. OGD, ^^^*p* < 0.05*ν*s. URB, ^&^*p* < 0.05*ν*s. AG, (*n* = 6). Magnificent: 200×, scale bar 20 *μ*m.

**Figure 3:** Effects of URB and AG on the tube formation and barrier function of BMECs subjected to OGD. (a) Representative the tube formation in each group. (b) Statistical analysis of length of tube formation. (c) The barrier property of BMECs monolayer was evaluated by TEER assay. (d) Effect of URB and AG on the barrier was also evaluated using EB albumin assays. ^∗^*p* < 0.05, *ν*s. Con, ^#^*p* < 0.05*ν*s. OGD, ^^^*p* < 0.05*ν*s. URB, ^&^*p* < 0.05*ν*s. AG, (*n* = 6). Magnificent: 100×, scale bar 100 *μ*m.

**Figure 4:** Effects of URB and AG on mitochondria ROS and inflammatory responses of BMECs subjected to OGD. (a) Representative histograms of flow cytometric evaluation of the cell-associated DCF-DA. (b) Quantitative analysis of cellular ROS levels. (c)–(e) Quantitative analysis of relative mRNA levels of TNF-*α*, IL-1*β*, and iNOS. (f) Standard protein curve. (g)–(i) Quantification of MDA level and activities of SOD and CAT in BMECs. ^∗^*p* < 0.05, *ν*s. Con, ^#^*p* < 0.05*ν*s. OGD, ^^^*p* < 0.05*ν*s. URB, ^&^*p* < 0.05*ν*s. AG, (*n* = 6).

**Figure 5:** Effects of URB and AG on mitochondrial membrane potential (MMP) of BMECs subjected to OGD. (a) Representative immunofluorescence of mitochondrial JC-1 in BMECs. (b) MMP as estimated by JC-1 red/green fluorescence intensity rate (FIR). ^∗^*p* < 0.05, *ν*s. Con, ^#^*p* < 0.05*ν*s. OGD, ^^^*p* < 0.05*ν*s. URB, ^&^*p* < 0.05*ν*s. AG, (*n* = 6). Magnificent: 400×, scale bar 50 *μ*m.

**Figure 6:** Effects of URB and AG on the distribution and expression of TJ proteins of BMECs subjected to OGD. (a) Representative ZO-1 (red) and Occludin (green) immunofluorescence staining in BMECs. (b, c) Quantitative analysis of relative fluorescence intensity of ZO-1 and Occludin. ^∗^*p* < 0.05, *ν*s. Con, ^#^*p* < 0.05*ν*s. OGD, ^^^*p* < 0.05*ν*s. URB, ^&^*p* < 0.05*ν*s. AG, (*n* = 6). Magnificent: 400×, scale bar 50 *μ*m.

**Figure 7:** Effects of URB and AG on activation of Nrf2 and TJ proteins of BMECs subjected to OGD. (a) Representative Nrf2 (red) immunofluorescence staining in BMECs. (b) Quantitative analysis of relative fluorescence intensity of Nrf2. (c) Representative Western blot bands of Nrf2, ZO-1, Occludin, and Claudin 5. (d)–(g) Quantitative analysis of the expressions of proteins. (h)–(k) The level of Nrf2, HO-1 after siRNA, URB, and AG treatment. ^∗^*p* < 0.05, *ν*s. Con/siNC, ^#^*p* < 0.05*ν*s. OGD, ^^^*p* < 0.05*ν*s. URB, ^&^*p* < 0.05*ν*s. AG, ^▽^*p* < 0.05*ν*s. siNrf2, (*n* = 3). Magnificent: 400×, scale bar 50 *μ*m.

**Figure 8:** Effects of URB and AG on apoptosis. (a) Representative TUNEL staining in BMECs. (b) Quantitative analysis of the apoptosis rate in TUNEL. (c, d) Cellar apoptosis was detected by Annexin V-FITC/PI flow cytometry analysis. ^∗^*p* < 0.05, *ν*s. Con, ^#^*p* < 0.05*ν*s. OGD, ^^^*p* < 0.05*ν*s. URB, ^&^*p* < 0.05*ν*s. AG, (*n* = 6). Magnificent: 200×, scale bar 20 *μ*m.

**Figure 9:** Possible mechanisms of URB and AG against OGD-induced BBB dysfunction and apoptosis. OGD inactivates the Nrf2 signaling, leading to the increase of proinflammatory factors and mitochondrial ROS. These cause a decrease in TJ protein expression and TJ degeneration in BMECs. The FAAH inhibitor URB597 and AG ameliorate BBB permeability and apoptosis by reducing oxidative stress and inflammation and activating Nrf2 signaling in OGD.

## Data Availability

The data that support the findings of this study are available from the corresponding authors (Qiao-Li Lv, lvqiaoli2008@126.com; Jian Hai, haijiandoct@zoho.com.cn) upon reasonable request.
